# The Effect of Health Education Combined with Personalized Psychological Nursing Intervention on Pregnancy Outcome of Pregnant Women with Gestational Diabetes Mellitus

**DOI:** 10.1155/2022/3157986

**Published:** 2022-03-19

**Authors:** Rubi He, Qiong Lei, Haibin Hu, Hui Li, Dongmei Tian, Zhicun Lai

**Affiliations:** Guangdong Women and Children Hospital, China

## Abstract

**Objective:**

To study the effect of health education combined with personalized psychological nursing intervention on pregnancy outcome of pregnant women with gestational diabetes mellitus (GDM).

**Methods:**

170 patients with GDM admitted to Guangdong Women and Children Hospital from January 2018 to December 2018 were selected as study subjects and randomly divided into two groups. During the period from diagnosis of GDM to termination of pregnancy, both groups were given routine education and routine examination, and the intervention group adopted health education combined with personalized psychological nursing interventions during pregnancy. The pregnancy weight, blood glucose index, compliance, disease awareness, self-adjustment management ability, satisfaction, and pregnancy outcome were measured before and after the intervention.

**Results:**

There were no statistically significant differences in pregnancy weight, fasting plasma glucose, and 2 h postprandial blood glucose between the two groups before intervention (*P* = 0.768, 0.605, and 0.762). After intervention, lower levels of the above indicators were obtained in the intervention group than in the control group (*P* < 0.001). The compliance and satisfaction with the intervention in the intervention group were significantly higher than those in the control group (*P* < 0.001). The intervention group had remarkably higher disease awareness rate and self-psychological adjustment and management ability than the control group (*P* < 0.001). Better pregnancy outcomes were observed in the intervention group compared with the control group (*P* < 0.001).

**Conclusion:**

For patients with GDM, health education combined with personalized psychological nursing on the basis of the conventional nursing can effectively control patients' condition and ensure a better pregnancy outcome, which merits widespread promotion.

## 1. Introduction

Gestational diabetes mellitus (GDM) is a disease in which normal glucose metabolism before pregnancy develops into a diabetic condition during pregnancy [1, 2], which is a common complication in women during pregnancy. In recent years, its incidence rate has witnessed an upward trend, and it can trigger symptoms such as premature birth, rupture of membranes, and postpartum hemorrhage, which takes a toll on the health of the patients and fetuses [3]. The proper control of blood glucose can mitigate the influence of blood glucose fluctuation on mothers and infants. Studies have shown that standardized health education for gestational diabetes can significantly improve patients' self-management ability while reducing their blood glucose levels [4, 5]. It can also help control the intake of sugars and lipids in the diet. With nondrug therapy, 80% of GDM patients' blood glucose can be controlled within an ideal range [6], which serves to improve the pregnancy outcome [7]. Herein, we identified patients with GDM who were enrolled in Guangdong Women and Children Hospital from January 2018 to December 2018 to examine the efficacy of health education combined with personalized psychological nursing intervention on them. The detailed report results are as follows.

## 2. Materials and Methods

### 2.1. General Information

A total of 170 patients with GDM admitted to Guangdong Women and Children Hospital from January 2018 to December 2018 were selected as research subjects. The selected patients were randomly divided into two groups with 85 patients in each group. In the control group, age is 20~40 years old, with an average age of 27.6 ± 2.5 years; there were 30 cases of primipara and 45 cases of multipara; gestational weeks are 24 to 38 weeks with an average of 28.3 ± 4.4 weeks; BMI is 16~29 kg/m^2^ with a mean value of 22.0 ± 5.9 kg/m^2^. In the intervention group, age is 20~38 years old, with an average age of 27.3 ± 3.0 years; there were 23 cases of primipara and 52 cases of multipara; gestational weeks are 23 to 38 weeks with an average of 28.4 ± 4.7 weeks; BMI is 16~29 kg/m^2^ with a mean value of 22.1 ± 5.9 kg/m^2^. The two groups showed no great disparity in terms of general information (*P* > 0.05).

Inclusion criteria (available at the same time) were as follows: (1) patients who meet the diagnostic criteria of WHO (2012) for GDM [8], (2) patients with single pregnancy, (3) patients without a history of diabetes before pregnancy, (4) patients with regular birth inspection, (5) patients with communication ability, and (6) patients who voluntarily participated in the study and signed the informed consent form.

Exclusion criteria (with one) were as follows: (1) patients with poor compliance or noncooperation or who were unwilling to continue the experiment during the study, (2) patients with serious complications or comorbidities, and (3) patients who have participated in other clinical investigations.

This study was approved by the ethics committee of our hospital, and all patients signed informed consent.

### 2.2. Methods

#### 2.2.1. Conventional Measures

During the period from the diagnosis of GDM to the termination of pregnancy, the two groups were given routine education and routine examination. Health guidance was given from the nurses in charge, and the patients were instructed to receive regular detection of blood glucose, control diet, and perform proper exercises. (1) Routine nursing. One-to-one education was provided to the patients and their families for a better understanding of the cause and harm of GDM, and the patients were encouraged perform proper exercises. 30 minutes of moderate intensity exercise every day could reduce postprandial blood glucose level. The patients were also guided in self-detection of blood glucose using a blood glucose meter. The daily postprandial test results were recorded and reported the nurses in charge. After analysis, the diet and exercise plan of the patients on the next day were timely adjusted. (2) Dietary guidance. The patients were instructed to adopt a low-fat, high-fiber, and low-glycemic diet. (3) Psychological intervention. Psychologists regularly carried out psychological counseling for patients to reduce the incidence of disease exacerbation due to anxiety, fear, and other negative emotions. (4) Discharge instructions. After discharge, a psychological follow-up was conducted to observe the psychological changes in the patients with timely guidance provided.

#### 2.2.2. Health Education Combined with Personalized Psychological Nursing Interventions during Pregnancy

On the basis of routine measures, the intervention group adopted health education combined with personalized psychological nursing interventions. (1) A health education team was set up, including one endocrinologist, one obstetrician, one pharmacist, one nutritionist, one psychological consultant, one maternal, one child specialist nurse, and three diabetes specialist nurses. Obstetricians and diabetes nurses were responsible for the unified training of the team members. The training contents were referred to the 2014 guidelines for the diagnosis and treatment of pregnancy with diabetes [9]. Considering the principles, content and process of structured intervention, research scheme, data collection and analysis, scale selection and use, GDM management, behavioral intervention, structured education curriculum, communication skills were included. (2) The health education group teaching method was implemented, with the participation of pregnant women with GDM and their families. The patients recorded the results of home blood glucose detection, shared their diet and exercise experience. With refer to guidelines for diabetes, six relevant courses were prepared for the patients, including basic knowledge of gestational diabetes, nutrition and exercise guidance during pregnancy, safe medication during pregnancy, blood glucose control and self-monitoring, psychological stress and coping, and postpartum follow-up guidance for gestational diabetes. The teaching forms included PPT, pictures, cartoons, short videos, health education prescription, and self-management manual. The team was responsible for providing online consultation and answering questions raised by the patients. According to the patients' conditions, readily comprehensible contents were provided to meet the health education needs of the patients. One-to-one online communication was also conducted through the WeChat group to further eliminate the patients' questions. When blood glucose reached the gestational control standard (fasting or preprandial blood glucose ≤ 5.3 mmol/L or 2 h postprandial blood glucose (2hPG) ≤ 6.7 mmol/L), with starvation ketosis and blood glucose exceeding the gestational standard after increasing caloric intake, personalized drug therapy were implemented in a timely manner. To explain in detail the safety of pregnant women hypoglycemic drug knowledge, team members should also send exercise videos such as maternal health exercise, maternal ball exercise and pelvic floor function training method for the patients to address their concerns about exercise treatment. Personalized guidance were also added to regular exercise during pregnancy according to the physiological characteristics of different stages of pregnancy. (3) Personalized psychological nursing intervention during pregnancy was performed according to the patient's past medical history, family history, adverse pregnancy and childbirth history, life and diet, exercise, and sleep habits. Patient who had anxiety, depression, and other negative emotions were given special psychological intervention and counseling. Patients with bad living habits were educated and guided to develop a good living habit. Patients with unhealthy dietary habits were instructed to follow a healthy diet. Team members should also closely observe the psychological changes of pregnant women, actively inquire about their feelings, and promptly provide psychological counseling when necessary, to reduce their concerns on the disease and ensure a better cooperation with the nursing. Moreover, successful cases of GDM were introduced to enhance the confidence of the patients. Psychological counseling was also given to the patients' families, to provide the patients with more support.

### 2.3. Observational Index

The pregnancy weight, blood glucose index, compliance, disease awareness rate, self-psychological regulation management ability, satisfaction, and pregnancy outcome of the two groups were measured before and after the intervention. Compliance was determined according to the performance of patients in terms of diet, blood glucose detection, and exercise therapy. The disease awareness rate and self-psychological adjustment and management ability were investigated by self-made questionnaire in our hospital, with the score of 0~100 points. The higher the score, the better the result. A self-made questionnaire was used to survey satisfaction, with a score of 0~100 points, and the higher the score, the more satisfied it was: very satisfied: ≥90 points, satisfied: 70-89 points, and dissatisfied: <70 points. Intervention satisfaction = (number of patients with very satisfied + satisfied)/total number of cases∗100%.

### 2.4. Statistical Analysis

The data were analyzed by SPSS23.0 statistical software, and the counting data were expressed as % and tested by *χ*^2^; measurement data are expressed as *x* ± *s* and tested by *t*; *P* < 0.05 meant that the difference between the two groups was statistically significant.

## 3. Results

### 3.1. Pregnancy Weight and Blood Glucose Indicators

There was no significant difference in pregnancy weight, fasting blood glucose, and 2 h postprandial blood glucose between the two groups before intervention (*P* = 0.768, 0.605, and 0.762). After intervention, the above indicators of the intervention group were significantly lower than those of the control group (*P* < 0.001) (see Table 1).

### 3.2. Compliance

The compliance of the intervention group was significantly higher than that of the control group (*P* < 0.001), as shown in Table 2.

### 3.3. Disease Awareness Rate and Self-Psychological Adjustment and Management Ability

The disease awareness rate and self-psychological adjustment and management ability of the intervention group were significantly higher than those of the control group (*P* < 0.001) (see Table 3).

### 3.4. Satisfaction

The satisfaction of the intervention group was significantly higher than that of the control group (*P* < 0.001) (see Table 4).

### 3.5. Pregnancy Outcomes

The pregnancy outcomes of the intervention group were significantly higher than those of the control group (*P* < 0.001) (see Table 5).

## 4. Discussion

GDM is a very common and frequent disease, which is related to the abnormal glucose tolerance of pregnant women and the abnormal increase in blood glucose level after onset [10, 11]. It can induce lactic acidosis, hyperosmotic coma, renal failure, pregnancy-induced hypertension, heart failure, and other related complications, which pose a threat to both the health of the patients and the growth and development of the fetus. Currently, patients with GDM are mainly treated with hypoglycemic drugs in clinical practice [12]. However, insufficient understanding of GDM in some patients and the existence of negative emotions such as anxiety and depression may undermine the compliance of patients and the clinical efficacy [13–15]. The pathogenesis of GDM is very complex and has not yet been elucidated. It has been pointed out that GDM may be related to insulin resistance, genetic factors, adipocytes, and inflammatory factors [16]. Delayed or improper treatment may threaten the health of mother and fetus and trigger a cascade of complications, such as placental abruption, macrosomia, and premature delivery [17, 18], which highlights the importance of patients' psychological status during pregnancy. The existing multiple GDM interventions, such as personalized nutrition guidance and self-management education, can improve the level of self-management and effectively control blood glucose [19]. However, notwithstanding a certain effect of general education and dietary guidance during hospitalization, the efficacy may be compromised after discharge due to poor compliance [20]. Therefore, to ensure a better quality of life of patients, our hospital provides health education and psychological nursing intervention for related patients with gestational diabetes, especially strengthening health education during pregnancy, to further enhance the treatment efficacy.

Among 170 GDM patients admitted to Guangdong Women and Children Hospital care hospital, GDM patients were divided into two groups, with routine nursing intervention for the control group and health education combined with personalized psychological intervention based on conventional nursing for the intervention group. The results showed that there were no statistically significant differences in pregnancy weight, fasting plasma glucose, and 2 h postprandial blood glucose between the two groups before intervention (*P* = 0.768, 0.605, and 0.762). After intervention, the above indicators of the intervention group were significantly lower than those of the control group (*P* < 0.001). The compliance and satisfaction with intervention in the intervention group were significantly higher than those in the control group (*P* < 0.001), indicating that health education combined with personalized psychological intervention can significantly improve patients' compliance. It could further control the weight gain of GDM patients and improve the blood glucose index of patients, thus increasing their satisfaction with the intervention. The intervention group had remarkably higher disease awareness rate and self-psychological adjustment and management ability than the control group (*P* < 0.001). Personalized health education could strengthen patients' understanding of GDM disease and improve patients' positive awareness of GDM. Better pregnancy outcomes were observed in the intervention group compared with the control group (*P* < 0.001). According to the results, nutrition and behavior intervention should be strengthened, and the mobile glucose health management platform should be established to realize the change of GDM patients' blood glucose management mode from informationized in-hospital blood glucose management to out-of-hospital blood glucose management mode, so as to improve patients' self-measurement blood glucose compliance. Furthermore, the establishment of a health education team contributes to a more convenient nursing intervention through the WeChat group, telephones, and other approaches to quickly solve patients' questions without the limit of time and space, as compared to traditional follow-up visits.

In conclusion, for patients with GDM, health education combined with personalized psychological nursing on the basis of the conventional nursing can effectively control patients' condition and ensure a better pregnancy outcome, which merits widespread promotion.

## Figures and Tables

**Table 1:** Comparison of pregnancy weight and blood glucose indicators.

Groups	2 h postprandial blood glucose (mmol/L)		Fasting plasma glucose (mmol/L)		Pregnancy weight	
	Before the intervention	After the intervention	Before the intervention	After the intervention	Before the intervention	After the intervention
Control group	7.67 ± 0.67	5.78 ± 0.67	6.27 ± 1.48	4.76 ± 0.67	54.28 ± 6.84	66.27 ± 3.68
Intervention group	7.73 ± 1.75	6.77 ± 0.78	6.39 ± 1.54	5.47 ± 0.83	54.60 ± 6.95	69.71 ± 4.42
*t*	0.4046	2.0364	0.3381	2.2203	0.2960	2.1073
*P*	0.768	<0.001	0.605	<0.001	0.762	<0.001

**Table 2:** Comparison of compliance.

Groups	According to exercise therapy		Cooperating with blood glucose monitoring		Eating according to the dietary requirements of GDM	
	Compliance (%)	Noncompliance (%)	Compliance (%)	Noncompliance (%)	Compliance (%)	Noncompliance (%)
Control group	80 (94.11)	5 (5.89)	82 (96.47)	3 `(3.53)	80 (94.11)	5 (5.89)
Intervention group	62 (72.94)	23 (27.06)	59 (69.41)	26 (30.59)	62 (72.94)	23 (27.06)
*χ* ^2^	13.850		21.990		13.850	
*P*	<0.001		<0.001		<0.001	

**Table 3:** Comparison of disease awareness rate and self-psychological adjustment and management ability.

Groups	Disease awareness rate	Self-psychological adjustment and management ability
Control group	96.13 ± 1.33	93.10 ± 3.32
Intervention group	83.34 ± 2.27	82.10 ± 3.32
*t*	44.820	21.600
*P*	<0.001	<0.001

**Table 4:** Comparison of satisfaction.

Groups	Very satisfied (%)	Satisfied (%)	Dissatisfied (%)	Satisfaction rate (%)
Control group	60 (70.59)	23 (27.06)	2 (2.35)	97.65
Intervention group	37 (43.53)	46 (36.47)	17 (20.00)	80.00
*χ* ^2^				13.330
*P*				<0.001

**Table 5:** Comparison of pregnancy outcomes.

Groups	Macrosomia (%)	Polyhydramnios (%)	Preterm birth (%)	Neonatal asphyxia (%)	Other (%)
Control group	7 (8.00)	7 (8.00)	9 (10.67)	7 (8.00)	8 (9.33)
Intervention group	0 (0.00)	2 (2.67)	2 (2.67)	2 (2.67)	2 (2.67)
*χ* ^2^					26.820
*P*					<0.001

## Data Availability

The data used to support the findings of this study are available from the corresponding author upon request.
